# Clinical Effect and Aesthetic Observation of All-on-4 Immediate Loading Implant Denture in Severe Periodontitis

**DOI:** 10.1155/2021/3120260

**Published:** 2021-08-20

**Authors:** Zhe Cheng, Wanlai Zheng

**Affiliations:** ^1^Songyang Yijia Dental Clinic, Lishui 323400, Zhejiang Province, China; ^2^Department of Functional Examination, Lishui People's Hospital, Lishui 323000, Zhejiang Province, China

## Abstract

**Objective:**

To explore the clinical effect and aesthetics of All-on-4 immediate loading implant denture in severe periodontitis.

**Methods:**

Totally, 60 patients with dentition loss caused by severe periodontitis who were admitted to our hospital from February 2017 to February 2019 were selected. The patients were randomly divided into the observation group (*n* = 30) and the control group (*n* = 30) according to different restoration methods. The control group was used in traditional implant restoration treatment, and the observation group was used in All-on-4 immediate loading implant denture restoration. The clinical effect, periodontal index, aesthetic effect, and complications of the two groups were compared, and the levels of serum leptin (LEP), tumor necrosis factor-*α* (TNF-*α*), C-reactive protein (CRP), and interleukin-6 (IL-6) were measured.

**Results:**

The total effective rate of the observation group (83.33%) was higher than that of the control group (60.00%) (*P* < 0.05). After treatment, the plaque index, gingival sulcus bleeding index, and depth of exploration of the two groups were lower than those before treatment (*P* < 0.05), and there was no significant difference between the two groups (*P* > 0.05). After treatment, the serum LEP, TNF-*α*, CRP, and IL-6 in both groups were lower than before treatment, and the serum LEP, TNF-*α*, CRP, and IL-6 in the observation group were lower than that in the control group (*P* < 0.05). The aesthetic rate of teeth in the observation group (90.00%) was higher than that in the control group (66.67%) (*P* < 0.05). There was no significant difference in the total incidence of complications between the two groups (*P* > 0.05).

**Conclusion:**

All-on-4 immediate loading implant denture has a good effect in the treatment of severe periodontitis, which is conducive to maintaining periodontal health, reducing the level of inflammation, improving aesthetics, and has high safety.

## 1. Introduction

Periodontitis is a chronic inflammation of periodontal supporting tissue caused by plaque, calculus, and other factors, which has become one of the common oral diseases [1]. The early symptoms of this disease are not obvious, but with the progress of the disease, there may occur loosening and shedding of teeth, soft tissue inflammation, alveolar bone absorption, and other symptoms. Some patients have developed into severe periodontitis [2]. According to the research survey, in 2010, the incidence of severe periodontitis was about 11% among people over 15 years old in the world, the incidence of severe periodontitis was about 12.1%–16.1% in China, and the incidence increased with the increase in age and ranking sixth among the global epidemic diseases [3]. Patients with severe periodontitis usually have heavy alveolar bone resorption and large distance between upper and lower jaws. Most patients may develop dentition loss, which has adverse effects on chewing, pronunciation function, and appearance [4]. With the continuous development of dental implant technology, implant restoration has become an effective treatment for dentition loss. In 2003, Maló et al. [5, 6] proposed the All-on-4 immediate loading planting scheme. This method is a repair method in which 4 implants are placed into the jaw bone, and restoration can be fixed on the same day. It has been widely used at home and abroad. The All-on-4 immediate loading implant technology has been carried out in our hospital for many years. In this study, through summarizing the rich clinical experience in our department, the efficacy of All-on-4 immediate loading implant denture in severe periodontitis and its influence on tooth aesthetic performance were discussed, to provide clinical reference.

## 2. Materials and Methods

### 2.1. Research Object

Totally, 60 patients with dentition loss caused by severe periodontitis who were admitted to our hospital from February 2017 to February 2019 were selected. Among them, there were 26 males and 34 females with an average age of (37.71 ± 4.72) years (range, 22–55 years). The patients were randomly divided into the observation group (*n* = 30) and the control group (*n* = 30) according to different restoration methods. There were no significant differences in general data between the two groups (*P* > 0.05), as shown in Table 1. This study has been approved by the ethics committee. All selected patients were informed of the purpose, method, and possible risks of the study and signed an informed consent.

#### 2.1.1. Inclusion Criteria

Inclusion criteria were as follows: age 18–65 years; met the diagnostic criteria for severe periodontitis; missing or remaining teeth should not be retained; alveolar bone resorption of the affected tooth reaches 1/2 to 1/3 of the root length, degree II to III looseness; the patients were in good condition and could tolerate the operation; some patients were accompanied by other diseases such as cardiovascular system, digestive system, endocrine system, and other diseases, but their conditions were under control, and according to the general condition of the patients, the implant restoration had no effect on their vital signs; fasting blood glucose <8.8 mmol/L; bone mass below the root tip >3 mm, and the four-wall bone plate of the extraction socket were relatively complete.

#### 2.1.2. Exclusion Criteria

Patients were accompanied by severe systemic diseases, but the condition had not been controlled; osteoporosis; night bruxism or dental occlusion disorder; lack of initial stability after implant placement, unable to complete immediate weight bearing; mental illness; uncontrolled blood sugar <8.8 mmol/L or blood pressure >140/90 mmHg; smoking more than 10 cigarettes/day or alcoholism (drinks almost every day and the average daily amount of alcohol equivalent to white spirit >200 g); and pregnant or lactating women.

### 2.2. Research Methods

Both groups were treated with conventional inflammation. The patients were treated with supragingival scaling, subgingival scaling, and root surface leveling. Patients were given cefuroxime axetil 500 mg, 2 times/d, the treatment lasted for 2 weeks, individual patients with deep periodontal pockets could be treated with curettage of the inner wall of the pocket to control periodontal inflammation. Preoperative evaluation was performed before treatment; inform the patients of their tooth condition, treatment procedures, and possible phenomena after treatment. Oral tomography and CBCT were taken to assess the bone mass and bone condition of the patient. The system and model of “All-on-4” implant were defined, and the position, axial direction, diameter, and length of the implant were determined by computer simulation, and the jaw position relationship was determined. Severe periodontal disease teeth with poor prognosis were extracted before operation, and the periodontal condition of other remaining teeth was controlled stably.

The control group was treated with traditional planting restoration technology. The unretainable teeth were extracted; after 3 months, implant implantation was performed. The panorama of the whole mouth was taken before the operation. The dentition loss and jaw position relationship were observed. The reasonable operation plan was formulated. 3–6 months after the operation, the second-stage operation was performed. Patients were instructed to maintain oral hygiene and review regularly.

The observation group was treated with used All-on-4 immediate loading implant denture restoration. Chlorhexidine solution was used to disinfect the whole mouth, lidocaine was used for local infiltration anesthesia, the teeth that could not be retained were extracted, and the granulation tissue in the tooth socket was scraped, and the alveolar bone was exposed in the field of vision. The position of the implants was clarified, and under the guidance of the digital guide, 4 implants were implanted using the Speedy Implant System from Sweden Nobel company. The single-jaw screw-retained one-piece fixed bridge supported by 4 implants was used. The 2 implants in the anterior part of the jaw were implanted vertically, and the 2 implants in the posterior part of the jaw were implanted at an angle, implant torque >0.35 (N·m) to ensure the initial stability of the implant. The multifunctional abutment was installed, the panorama of the whole mouth was taken to determine the position of implant and abutment, and the wound was sutured routinely. One hour after implantation was completed, the impression was made, and the temporary restoration made of polyacrylate material was completed. The temporary restoration was designed with short dental arch and only restored to the second premolar or reduced one premolar to the first molar and adjusted the occlusal relationship. Within 48 hours, the temporary restorations with screw retention as the retention method were worn. Instruct patients to keep oral hygiene, avoid eating hard food, anti-inflammatory treatment for 3–5 days, and review regularly. Six months to 12 months after the operation, the implant supported fixed denture was made according to the occlusal condition and patients' wishes. The types of permanent restorations include overdentures supported by implants, polyacrylate restorations supported by cobalt-chromium alloy stents, and porcelain restorations supported by metal stents. The average follow-up time for all patients was 12 months.

Postoperative oral maintenance was performed for the two groups: patients in both groups were instructed to use dental floss daily to clean the tissue surface of the restoration after surgery, at the same time, the patients were instructed to cooperate with the flushing device and interdental brush, pay attention to oral hygiene, and avoid long-term consumption of hard objects.

### 2.3. Observation Index

#### 2.3.1. Efficacy Evaluation Criteria

After treatment, the therapeutic effects of the two groups were evaluated. Effective: no pain and periodontal inflammation, no loosening or shedding of the implant, no progressive bone resorption, and X-ray showed no low-density transmission area around the implant; improvement: occasional pain and periodontal inflammation, slight implant loosening, but no shedding, no progressive bone resorption, and X-ray showed no low-density transmission area around the implant; ineffective: often accompanied by pain and periodontal inflammation, implant serious loosening or shedding, progressive bone resorption, and X-ray showed that the implant had a low-density area of alveolar bone. Total effective rate = (effective + improvement) cases/total cases × 100%.

#### 2.3.2. Periodontal Index

Before and after treatment, full-mouth periodontal examination was performed, and periodontal index was detected at 6 sites of mesial, median, and distal buccal and lingual surface of each tooth: plaque index (PLI), gingival sulcus bleeding index (SBI), and probing depth (PD) [7–9]. The plaque display agent was used in PLI, and the patients gargled the plaque display agent for 2 minutes. The red attachment sites on the teeth were observed. 0 point: no plaque, 1 point: a small amount of plaque can be scraped from the side of the probe tip, 2 points: medium plaque can be scraped from the side of the probe tip, and 3 points: a large amount of soft dirt can be scraped from the side of the probe tip. SBI was detected by periodontal probe with a force of 0.2 N along the gingival margin of the implant, 0 point: no bleeding during the probing, 1 point: punctate bleeding, 2 points: linear bleeding in the gingival sulcus, and 3 points: blood overflowing from the gingival sulcus. PD was detected by periodontal probe with a force of 0.2 N to measure the distance from the gingival margin to the bottom of the pocket or the bottom of the gingival sulcus. All measurements were performed by the same operator.

#### 2.3.3. Laboratory Indexes

Before and after treatment, 7 mL of fasting venous blood was collected from the patient in the morning, centrifuged at 3000 r/min for 8 min, and enzyme-linked immunoassay was used to detect serum leptin (LEP), tumor necrosis factor-*α* (TNF-*α*), C-reactive protein (CRP), and interleukin-6 (IL-6) levels.

#### 2.3.4. Kay's Aesthetic Classification of Teeth

Six months after treatment, the aesthetic condition of the patients was evaluated: Class I: completed aesthetic structure; Class II: slight changed of aesthetic structure; Class III: the aesthetic results changed significantly; and Class IV: deformity. Total aesthetic rate = (class I + class II) cases/total cases × 100% [10].

#### 2.3.5. Complications

The incidence of complications in the two groups within 6 months after treatment was recorded, including gingival atrophy, pain in occlusion, oral infection, peri-implantitis, fracture of restoration, and other problems.

### 2.4. Statistical Methods

SPSS 22.0 software was used for analysis, measurement data were expressed as mean ± standard deviation, and *t*-test was used to analyze the comparison. Count data were expressed as a ratio, and χ^2^-test was used to analyze the comparison. *P* < 0.05 was statistically significant.

## 3. Results

### 3.1. Comparison of Clinical Efficacy between the Two Groups

The total effective rate of the observation group (83.33%) was higher than that of the control group (60.00%) (*P* < 0.05), as shown in Figure 1.

### 3.2. Comparison of Periodontal Index between the Two Groups

Before treatment, there was no difference between the two groups of periodontal indexes of PLI, SBI, and PD (*P* > 0.05). After treatment, the PLI, SBI, and PD of the two groups were lower than those before treatment (*P* < 0.05), and there was no significant difference between the two groups (*P* > 0.05), as shown in Figure 2.

### 3.3. Comparison of Laboratory Indexes between the Two Groups

Before treatment, there was no difference between the two groups of serum LEP, TNF-*α*, CRP, and IL-6 (*P* > 0.05). After treatment, the serum LEP, TNF-*α*, CRP, and IL-6 in both groups were lower than before treatment, and the serum LEP, TNF-*α*, CRP, and IL-6 in the observation group were lower than that in the control group (*P* < 0.05), as shown in Figure 3.

### 3.4. Comparison of Kay's Aesthetic Classification of Teeth between the Two Groups

The aesthetic rate of teeth in the observation group (90.00%) was higher than that in the control group (66.67%) (*P* < 0.05), as shown in Figure 4.

### 3.5. Comparison of Complications between the Two Groups

There was no significant difference in the total incidence of complications between the two groups (*P* > 0.05), as shown in Figure 5.

### 3.6. Typical Cases of Observation Group

A typical patient, male, 55 years old, with severe periodontitis leading to dentition defect, low mandibular alveolar ridge, and poor retention of removable denture, has never been used. After communicating with the patient, the patient agreed to perform mandibular All-on-4 immediate loading restoration. After 12 months of restoration, the effect was good, the implant was not loose and fell off, and the aesthetics was significantly improved, as shown in Figure 6.

## 4. Discussion

Severe periodontitis is one of the common diseases in stomatology, and its main symptoms are tooth loosening, tooth loss, and alveolar bone resorption, which usually leads to the loss of dentition and affects the daily life and physical and mental health of patients [11]. Therefore, it is of great significance to take reasonable and effective measures to solve the problems of dentition loss and alveolar bone resorption [12]. All-on-4 immediate loading implant can be implanted into 4 implants and can be put into the implant support restoration immediately after operation, which can achieve the purpose of immediate loading implant, and has beneficial effects such as easy operation, shortening the course of treatment, and quick recovery [13, 14]. To further search for safe and effective implant restoration methods, we applied the traditional implant repair technology and All-on-4 immediate loading implant technology to the patients with dentition loss and observed the clinical effect of both. The experience was summarized as follows.

Our hospital has rich clinical experience in dental implant technology. According to the principle of safe, effective, and beautiful, we believe that All-on-4 immediate loading implant technology has many advantages. It is easy to operate, fast to perform function, consistent with the biomechanical characteristics of the tooth, high implant stability, can avoid the absorption of alveolar soft tissue, and has a good effect [15]. Our physicians found that the total effective rate of the observation group was higher than that of the control group, and there was no significant difference in periodontal indexes between the two groups. The results showed that both All-on-4 immediate loading implant and traditional implant restoration are beneficial to maintaining periodontal health, and All-on-4 immediate loading implant has more significant effect on patients with severe periodontitis. We believe that the possible reason is that the traditional implant restoration technology has a high curative effect (60.00%), which can significantly improve the retention of the covered denture, improve the comfort of the patient, and have a positive effect on daily life and aesthetics. However, this technique can only be implemented 3 months after the extraction of the affected teeth, and the second-stage treatment can be implemented 3–6 months after the implantation, which has certain limitations such as long course of treatment and poor chewing function. At the same time, a long course of treatment will lead to severe discomfort of patients, and inadequate daily maintenance may cause inflammation and damage of periodontal tissue [16]. The All-on-4 immediate loading implant surgery only needs one operation, and it is easy to operate and less traumatic, which can reduce the adverse impact of the lack of teeth on the daily life of patients [17, 18]. The All-on-4 immediate loading implant technology cleverly avoid the nerve distribution of the maxillary sinus and inferior alveolar through the preoperative detailed design and implanted the implant into the relatively dense place of the mandibular bone, so that the bone mass of the anterior mandible can be fully utilized. At the same time, this technology can greatly reduce the length of the cantilever beam of the denture, thereby reducing the damage to the patient and improving the accuracy of implantation [19]. The All-on-4 immediate loading implant technology is helpful to stimulate the formation of new bone in the stress concentration area, rationally distribute the bone trabecula around the implant according to the form of force, and promote the reconstruction of bone tissue. In addition, it can ensure the amount of bone around the implant, form a good gingival papilla shape, and avoid the phenomenon of “black triangle”.

As a hormone secreted by adipose tissue, LEP can reflect the level of inflammation in the body and is a key factor leading to host infection and the production of proinflammatory factors. At the same time, periodontitis is mainly caused by G-anaerobe infection, and its endotoxin lipopolysaccharide can stimulate the secretion of inflammatory factors such as TNF-*α*, CRP, and IL-6, which increase the inflammation level of periodontal tissues [20, 21]. All-on-4 immediate loading implant technology can effectively improve the oral environment of patients with severe periodontitis and reduce the level of inflammation. The results of this study suggested that the serum levels of LEP, TNF-*α*, CRP, and IL-6 were significantly decreased in the observation group. In this study, after restoration, the observation group had a higher aesthetic rate of teeth. The All-on-4 immediate loading implant technology design an aesthetic and reasonable plan according to the actual situation of the patients before restoration, which could reduce the tooth inclination caused by implant movement, ensure the smoothness of the alveolar, make the alveolar ridge more full, and improve the aesthetic performance. In addition, there was no significant difference in the total incidence of complications between the two groups. The results showed that the All-on-4 immediate loading implant technology is safe in the treatment of severe periodontitis. In our opinion, it is necessary to grasp the basic situation of patients clinically, strictly control the indications, ask patients to have regular review after surgery, pay attention to oral hygiene, maintain good living habits, and properly care for the denture, so as to reduce the incidence of complications.

All-on-4 immediate loading implant technology has become a commonly surgical method in clinical practice, which plays a key role in implant repair. However, it should be noted that this method is not suitable for all patients with severe periodontitis and has high surgical requirements. For example, the All-on-4 immediate loading implant technology should not be used when the cantilever of denture is too long or the occlusal strength is too high. Therefore, based on the summary of many years of prosthetic experience, we think that the surgeons should evaluate the bone condition and implant stability of the patients before operation, strictly follow the operational specification during operation, and maintain the periodontal health of the implants after operation, so as to meet the ideal needs of patients.

## 5. Conclusion

In summary, All-on-4 immediate loading implant denture has a good effect in the treatment of severe periodontitis, which is conducive to maintaining periodontal health, reducing the level of inflammation, improving aesthetics, and has high safety. The shortcomings of the study are that the sample size is small, and the follow-up time is short. It is necessary to expand the sample size and extend the follow-up time in future study, so as to observe the long-term efficacy.

## Figures and Tables

**Figure 1:** Comparison of clinical efficacy between two groups. Note: compared with the control group, ^*∗*^*P* < 0.05.

**Figure 2:** Comparison of periodontal index between two groups. Note: compared with before treatment, ^#^*P* < 0.05.

**Figure 3:** Comparison of laboratory indexes between the two groups. Note: compared with the control group, ^*∗*^*P* < 0.05; compared with before treatment, ^#^*P* < 0.05.

**Figure 4:** Comparison of Kay's aesthetic classification of teeth between the two groups. Note: compared with the control group, ^*∗*^*P* < 0.05.

**Figure 5:** Comparison of complications between the two groups of patients.

**Figure 6:** Typical cases of observation group: (a) before implant restoration, the jaw and periodontal conditions of the patients; (b) imaging examination of mandibular All-on-4 immediate loading restoration; (c) temporary restoration after immediate implantation; (d) imaging examination after 12 months of All-on-4 permanent repair; (e) intraoral pictures after the permanent restoration was put on for 12 months.

**Table 1:** Comparison of general data between the two groups (*n*, %, $\bar{x}$ ± *s*).

Group	Gender		Average age (years)	Average course of disease (months)	Missing tooth position		Tooth looseness	
	Male	Female			Loss of upper anterior teeth	Loss of lower anterior teeth	Degree II	Degree III
Control group (*n* = 30)	12 (40.00%)	18 (60.00%)	38.19 ± 4.47	6.29 ± 1.09	21 (70.00%)	9 (30.00%)	11 (36.67%)	19 (63.33%)
Observation group (*n* = 30)	14 (46.67%)	16 (53.33%)	37.23 ± 4.81	6.32 ± 1.02	18 (60.00%)	12 (40.00%)	9 (30.00%)	21 (70.00%)
χ^2^*/t* value	0.271		0.801	0.110	0.659		0.300	
*P* value	0.602		0.426	0.912	0.417		0.584	

## Data Availability

The data used during the current study are available from the corresponding author.

## References

[1] Helal O., Göstemeyer G., Krois J., Fawzy El Sayed K., Graetz C., Schwendicke F. (2019). Predictors for tooth loss in periodontitis patients: systematic review and meta-analysis. *Journal of Clinical Periodontology*.

[2] Yan X., Wu Z., Wang B. (2020). Involvement of cathepsins in innate and adaptive immune responses in periodontitis. *Evidence-based Complementary and Alternative Medicine: eCAM*.

[3] Kassebaum N. J., Bernabé E., Dahiya M., Bhandari B., Murray C. J. L., Marcenes W. (2014). Global burden of severe periodontitis in 1990-2010. *Journal of Dental Research*.

[4] Slots J. (2020). Primer on etiology and treatment of progressive/severe periodontitis: a systemic health perspective. *Periodontology 2000*.

[5] Maló P., Rangert B., Nobre M. (2005). All-on-4 immediate-function concept with Brånemark System implants for completely edentulous maxillae: a 1-year retrospective clinical study. *Clinical Implant Dentistry and Related Research*.

[6] Maló P., Rangert B., Nobre M. (2003). “All-on-Four” immediate-function concept with brånemark system implants for completely edentulous mandibles: a retrospective clinical study. *Clinical Implant Dentistry and Related Research*.

[7] Woelber J. P., Bremer K., Vach D. (2016). An oral health optimized diet can reduce gingival and periodontal inflammation in humans-a randomized controlled pilot study. *BMC Oral Health*.

[8] Monje A., Wang H.-L., Nart J. (2017). Association of preventive maintenance therapy compliance and peri-implant diseases: a cross-sectional study. *Journal of Periodontology*.

[9] Pei X. Y., He L., Ouyang X. Y. (2017). Proposing a novel, three-level definition of periodontitis using probing depth, clinical attachment loss and bleeding on probing: analysis of a rural Chinese population. *Chinese Journal of Dental Research*.

[10] Kay H. B. (2002). Classification of altered dental esthetics. *The International Journal of Periodontics & Restorative Dentistry*.

[11] Slots J. (2020). Life‐threatening pathogens in severe/progressive periodontitis: focal infection risk, future periodontal practice, role of the Periodontology 2000. *Periodontology 2000*.

[12] Manresa C., Sanz-Miralles E. C., Twigg J., Bravo M. (2018). Supportive periodontal therapy (SPT) for maintaining the dentition in adults treated for periodontitis. *Cochrane Database of Systematic Reviews*.

[13] Maló P., de Araújo Nobre M., Lopes A., Ferro A., Botto J. (2019). The All-on-4 treatment concept for the rehabilitation of the completely edentulous mandible: a longitudinal study with 10 to 18 years of follow-up. *Clinical Implant Dentistry and Related Research*.

[14] ELsyad M. A., Elgamal M., Mohammed Askar O., Youssef Al‐Tonbary G. (2019). Patient satisfaction and oral health‐related quality of life (OHRQoL) of conventional denture, fixed prosthesis and milled bar overdenture for All‐on‐4 implant rehabilitation. A crossover study. *Clinical Oral Implants Research*.

[15] Li S., Di P., Zhang Y., Lin Y. (2017). Immediate implant and rehabilitation based on All-on-4 concept in patients with generalized aggressive periodontitis: a medium-term prospective study. *Clinical Implant Dentistry and Related Research*.

[16] Chan M. H., Holmes C. (2015). Contemporary “All-on-4” concept. *Dental Clinics of North America*.

[17] Penarrocha-Diago M., Penarrocha-Diago M., Zaragozí-Alonso R., Soto-Penaloza D., On B. O. T. T. (2017). Consensus statements and clinical recommendations on treatment indications, surgical procedures, prosthetic protocols and complications following All-On-4 standard treatment. 9th Mozo-Grau Ticare Conference in Quintanilla, Spain. *Journal of Clinical and Experimental Dentistry*.

[18] Cucchi A., Vignudelli E., Franco S., Ghensi P., Malchiodi L., Corinaldesi G. (2019). Evaluation of crestal bone loss around straight and tilted implants in patients rehabilitated by immediate-loaded full-arch all-on-4 or all-on-6: a prospective study. *Journal of Oral Implantology*.

[19] Yilmaz B., Ozcelik T. B., McGlumphy E. (2015). Using the “final-on-four” concept to deliver an immediate metal-resin implant-fixed complete dental prosthesis. *The Journal of Prosthetic Dentistry*.

[20] Purnamasari D., Khumaedi A. I., Soeroso Y., Marhamah S. (2019). The influence of diabetes and or periodontitis on inflammation and adiponectin level. *Diabetes & Metabolic Syndrome: Clinical Research & Reviews*.

[21] Chen X., Wang L., He Z. (2020). Effects of xipayi mouth rinse combined with minocycline on localized aggressive periodontitis’ therapeutic effect and the levels of CRP, TNF-*α*, IL-6 in serum. *Annals of Palliative Medicine*.

